The article "PIWIL2 restrains the progression of thyroid cancer via interaction with miR-146a-3p" was retracted in 2025. Reason: lack of ethics approval or compliance.

# PIWIL2 restrains the progression of thyroid cancer via interaction with miR-146a-3p

**DOI:** 10.1186/s12902-023-01416-0

**Published:** 2023-08-29

**Authors:** Xiaoxiao Lu, Qingyun Zhu, Hong Du, Mingjun Gu, Xiangqi Li

**Affiliations:** 1 Department of Endocrinology and Metabolism, Punan Hospital, Pudong New Area, Shanghai, 200125 China; 2 Department of Intervention, Gongli Hospital, Naval Medical University, Shanghai, 200135 China; 3 Department of General Practice, Hudong Community Health Service Centre, Pudong New Area, Shanghai, 200129 China; 4 Department of Endocrinology and Metabolism, Gongli Hospital, Naval Medical University, Shanghai, 200135 China

**Keywords:** PIWIL2, miR-146a-3p, Thyroid cancer, Reproduction, Cell proliferation, Cell cycle, Apoptosis, Migration, Invasion

## Abstract

**Objective:**

The classical role of PIWIL2 is to regulate reproduction by binding to piRNA, but its tumor-related function has received increasing attention in recent years. This study aims to explore its role in the progression of thyroid cancer (TC).

**Methods:**

First, we measured and analyzed the levels of PIWIL2 and miR-146a-3p in TC tissue and adjacent tissues as well as several TC cell lines. We demonstrated the clinical significance of PIWIL2 and miR-146a-3p through the survival rate. Based on these results, we selected TPC-1 and KTC-3 cell lines for our cell experiments. We treated these cell lines with PIWIL2 lentivirus, PIWIL2 siRNA, miR-146a-3p mimic, or miR-146a-3p inhibitor and measured cell proliferation, cell cycle, apoptosis, migration, and invasion. We used PCR and Western blot to quantify the mRNA and protein levels of PIWIL2, while we used luciferase reporter assay and RNA binding protein immunoprecipitation to explore the relationship between miR-146a-3p and PIWIL2. Finally, we developed a xenograft tumor model to confirm the effects of the miR-146a-3p/PIWIL2 axis on TC progression in vivo.

**Results:**

We identified that PIWIL2 and miR-146a-3p exhibit opposite expression alterations in TC tissues and that PIWIL2 serves as a ‘sponge’ by adsorbing miR-146a-3p. Up-regulating PIWIL2 decelerated the proliferation, metastasis, and cell cycle progression of TPC-1 and KTC-3 cells, but accelerated the apoptosis of TC cells, while miR-146a-3p exhibited opposite effects. Finally, overexpressing PIWIL2 restrained the progression of TC in nude mice, which can be reversed by increasing miR-146a-3p expression. Inhibiting PIWIL2, on the other hand, promoted the progression of TC in vivo, which can be reversed by inhibiting miR-146a-3p.

**Conclusion:**

PIWIL2 may inhibit the progression of TC by sponging miR-146a-3p, providing new insights into the early treatment, recrudescence treatment, and metastasis treatment of TC.

The article "PIWIL2 restrains the progression of thyroid cancer via interaction with miR-146a-3p" was retracted in 2025. Reason: lack of ethics approval or compliance.

**Supplementary Information:**

The online version contains supplementary material available at 10.1186/s12902-023-01416-0.

## Introduction

P-element induced wimpy testis like 2 (PIWIL2), also known as cancer/testis antigen 80 (CT80), belongs to the Argonaute family of proteins [1]. Its primary function is to control reproduction by binding to piRNA, a newly discovered type of small RNA, in the testes [2]. However, increasing evidence suggests that it also plays a crucial role in cancer development [3]. Studies have shown that PIWIL2 may impact prostate cancer [4], cervical cancer [5], oral squamous cell carcinoma [6], and esophageal squamous cell carcinoma [7]. In a multiple transcriptome analysis, it was also found that PIWIL2-induced cancer stem cells showed significant alterations in the levels of small RNAs [8]. Additionally, distinct changes in PIWIL2 expression were observed in thyroid cancer (TC) [8]. However, the pathological role of PIWIL2 in TC is yet to be determined.

TC (Thyroid Cancer) is one of the most prevalent endocrine malignancies [9]. Despite having a better survival rate compared to other cancers, its incidence has been consistently increasing over the years [10, 11]. However, treating TC patients with recurrence and metastasis remains a challenge, and the mortality rate of advanced TC remains a significant concern. Therefore, it is crucial to investigate new therapeutic targets and the underlying mechanisms of TC development.

In this present study, we first measured and analyzed the levels of PIWIL2 and miR-146a-3p in both TC tissue and adjacent tissues. Following this, we conducted cellular and molecular assays to investigate the pathological role and underlying mechanism of PIWIL2 in TC at the cellular and nude mouse levels. Our findings suggest that PIWIL2 could inhibit TC development through the process of miR-146a-3p sponging. Consequently, we offer new insights into the role of PIWIL2, which differ from the commonplace function it carries out by binding to a piRNA in the process of reproduction.

## Materials and methods

### TC samples collection and examination

A total of 20 paired thyroid tumor and adjacent non-tumor tissue samples were collected from Punan Hospital between January and December 2020. The clinical information of these patients can be found in Supplementary Table S1. Informed consent was obtained from all patients and the research was approved and supervised by the Ethics Committee of Punan Hospital. All tissue samples were snap-frozen and stored at − 80 °C. The miRNA levels of PIWIL2 and miR-146a-3p in the thyroid cancer tissue and adjacent tissues were measured, and the correlation between them was analyzed. The protein expression of PIWIL2 in the thyroid cancer tissue and adjacent tissues was measured by Western blotting. The survival time of these 20 patients was monitored and recorded. They were divided into two groups based on the miRNA levels of PIWIL2 and miR-146a-3p, and the difference in survival rate between these two groups was analyzed. The results are presented in Fig. 1.

The article "PIWIL2 restrains the progression of thyroid cancer via interaction with miR-146a-3p" was retracted in 2025. Reason: lack of ethics approval or compliance.

**Fig. 1:** Expression of PIWIL2 and miR-146a-3p in TC tissues **(A)** The mRNA expression of PIWIL2 in TC tissues. GAPDH was used for normalization. **(B)** The mRNA expression of miR-146a-3p in TC tissues. RNU6B was used for normalization. **(C)** Linear regression and correlation analyses between the expression of miR-146a-3p and the expression of PIWIL2 in clinical TC specimens. **D, E.** The protein expression of PIWIL2 in TC tissues. GAPDH was used for normalization. **F.** The survival rate of patients divided by the miRNA levels of PIWIL2. **G.** The survival rate of patients divided by the miRNA levels of miR-146a-3p. *: P < 0.05. N = 20. TC: thyroid cancer

### Cell culture

The TPC-1, KTC-3, WRO, PDTC-1, SW579 and FTC-133 cell lines were obtained from the American Type Culture Collection (ATCC, USA), while the NTHY-ORI 3 − 1 cells (human normal thyroid follicular epithelial cells) were obtained from Aidingbao Biological Technology Development Company (Shanghai, China) and used as a control. TPC-1 cells were derived from human thyroid papillary carcinoma, KTC-3 cells from human anaplastic thyroid cancer, WRO cells from human dedifferentiated thyroid cancer, PDTC-1 cells from poorly differentiated thyroid carcinoma, SW579 cells from squamous thyroid cancer, and FTC-133 cells from human follicular thyroid carcinoma.The cells were cultured at 37 °C and 5% CO2. Briefly, cell lines were maintained in DMEM Medium (Hyclone, USA) or RPMI-1640 medium (Sigma, USA) supplemented with 10% (v/v) fetal bovine serum (FBS) (Gibco, USA), 100 IU/mL penicillin and 100 µg/mL streptomycin (Beyotime, Shanghai, China).

### Cell transfection

Greenseed Biotech (Shanghai, China) supplied the miR-146a-3p inhibitor, miR-146a-3p mimic, PIWIL2 lentivirus, and PIWIL2 siRNA which were then transfected into TPC-1 and KTC-3 cells according to the instructions of the Lipofectamine 3000 reagent (ThermoFisher, USA). TPC-1 and KTC-3 cells were incubated until they were 70% confluent and then transfected with either 50 nM of miR-146a-3p mimic or mimic NC, or 100 nM of miR-146a-3p inhibitor or inhibitor NC in accordance with the manufacturer’s protocol. For PIWIL2 lentivirus transducing unit infection, 1 × 10^5^ TPC-1 and KTC-3 cells were infected with 1 × 10^7^ lentivirus transducing units of PIWIL2 in the presence of 10 µg/ml polybrene as per the manufacturer’s protocol. An empty lentiviral vector was used as a negative control. The PIWIL2 siRNA was mixed with the transfection reagent at a ratio of 15 nmol RNA to 1 µl reagent and was incubated at room temperature for 15 min. The RNA/reagent complex was then added to wells with antibiotics-free culture medium and further treatment was carried out for 48 h. Cells were harvested for further experiments 24 h after transfection.

The article "PIWIL2 restrains the progression of thyroid cancer via interaction with miR-146a-3p" was retracted in 2025. Reason: lack of ethics approval or compliance.

### Cell proliferation assay

To assess cell viability, the MTT Cell Proliferation and Cytotoxicity Assay Kit (Beyotime, Shanghai, China) was utilized. The cells were seeded into 96-well plates (1 × 10^4^ cells per well) in triplicate and allowed to grow synchronously for 24 h in serum-free medium. Afterward, 10 µL MTT reagent was added to each well, and the cells were incubated for an additional 4 h in a humidified incubator (37 °C, 5% CO_2_). The supernatant was discarded, and 200 µL DMSO was added to dissolve the formazan. The OD value was then measured at 570 nm using a Synergy. H1 microplate reader (BioTek, USA). The viability of the Control group was defined as 100%, and the viability of non-treated cells and cells from other groups was calculated separately based on that value.

### Cell invasion assay

To detect cell invasion [12], TPC-1 cells (1 × 10^5^ cells/mL) were resuspended in 200 µL of FBS-free RPMI-1640 medium and plated into the top chamber of a Matrigel-coated Transwell containing 500 ng/ml. In the lower chamber, 600 µL of RPMI-1640 medium with 20% FBS (Gibco, USA) was added. After incubating for 24 h, methanol was used to immobilize the cells in the lower chamber at 4 °C for 30 min, and then they were stained with crystal violet for 20 min. The cell images were captured by randomly selecting five fields and counting using ImageJ software (National Institute of Health, Bethesda, MD, USA) after the cells were washed with PBS.

### RNA binding protein immunoprecipitation (RIP)

Before cross-linking with 0.01% formaldehyde for 15 min, TPC-1 and KTC-3 cells were washed. After centrifugation at 10,000 g for 10 min, the cell pellets were lysed with an ice-cold polysome lysis buffer consisting of 100 mM KCl, 5 mM MgCl2, 10 mM Hepes (pH 7.0), and 0.5% Nonidet P-40. The cells were then incubated with a RIP buffer containing protein A/G magnetic beads coated with anti-PIWIL2 antibody or negative control anti-IgG antibody (Abcam, Cambridge, MA, USA) overnight at 4 °C. The cells were subsequently exposed to Protein A Agarose for 1 h at 4 °C. RNA was then isolated and miR-146a-3p levels detected using RT-PCR.

The article "PIWIL2 restrains the progression of thyroid cancer via interaction with miR-146a-3p" was retracted in 2025. Reason: lack of ethics approval or compliance.

### Wound healing assay

For the wound healing test [12], TPC-1 cells were cultured overnight in six-well plates with 5 × 10^5^ cells per well. A wound was created in each well using a 200-µL pipette tip followed by culturing for 48 h. The healing distance was photographed before and after culturing, and the wound-healing rate was then calculated.

### Flow cytometry assay

To determine the cell apoptotic rate, we utilized an Annexin V-APC and 7-AAD kit (Keygen, China) in a flow cytometry assay. Apoptosis of TC cells was induced by treating them with cisplatin (Beyotime, Shanghai, China) at a final concentration of 20 µM for 12 h. Cells were harvested and suspended in a binding buffer (5 × 10^5^ cells/mL) before being stained with Annexin V-APC and 7-AAD. The apoptotic cells were then analyzed using a FACScan® flow cytometry machine (BD Biosciences, USA).

### Cell cycle analysis

Each group of cells was inoculated into 6-well plates and cultured until their concentration reached 30-50%. The cells were then collected, washed with PBS buffer, and fixed in 70% ethanol at 4 °C overnight. RNA was removed from the cells using RNase A at 37 °C for 30 min. The fixative was then washed off, and 300 µL of PI/RNase A staining working solution was added to each well. The cells were incubated at room temperature in the dark for 60 min. Finally, the cell cycle distribution was analyzed by using ModFit LT software (Verity Software House, Topsham, ME) [12]. This experiment was repeated three times for accuracy.

### Luciferase reporter assay

The TargetScan web-based tool (http://www.targetscan.org/vert_71/) [13] was used to predict the binding site between miR-146b-3p and the 3’-UTR of PIWIL2. The fragment of PIWIL2 was amplified through PCR and cloned to the downstream of the Renilla psiCHECK2 vector (Promega, USA) [14], resulting in wt-PIWIL2. In order to generate the PIWIL2 mutant reporter, the seed region of the PIWIL2 was mutated to remove all complementarity to nucleotides 2–7 of miR-146a-3p, resulting in mut-PIWIL2. HEK293 cells (ATCC, USA) were seeded in a 24-well plate and co-transfected with the designated vectors and miR-146a-3p mimics or control mimics. Luciferase assays were conducted 48 h after transfection using the Dual Luciferase Reporter Assay System (Promega, USA). Renilla luciferase activity was normalized to Firefly luciferase activity in each transfected well.

### Real-time quantitative polymerase chain reaction (RT-PCR)

Total RNA was extracted using the Trizol reagent (Invitrogen, USA) according to the manufacturer’s instructions. MiRNA-specific primers were used for reverse transcription of the total RNA, and the miScript Reverse Transcription kit (Qiagen, Germany) was used for miRNA qRT-PCR. We used RNU6B expression as an endogenous control. To detect mRNA expression, we used the One Step SYBR PrimeScript RT-PCR kit (Takara Biotechnology, China) following the protocol. We performed the reaction using the ABI PRISM 7500 Real-Time PCR system (ThermoFisher, USA), with incubation at 42 °C for 5 min, 95 °C for 10 s, followed by 40 cycles of 95 °C for 5 s, 55 °C for 30 s, and 72 °C for 30 s. We repeated each independent experiment three times. We used GAPDH expression as an endogenous control. We analyzed relative fold changes using the 2^−ΔΔCt^ value method. Supplementary Table S2 lists the primers used in this study.

The article "PIWIL2 restrains the progression of thyroid cancer via interaction with miR-146a-3p" was retracted in 2025. Reason: lack of ethics approval or compliance.

### Absolute quantification of PIWIL2 and miR-146a-3p copies

In the TPC-1 and KTC-3 cells, the absolute PIWIL2 and miRNA transcript abundance was quantitated using the standard curve method. Afterwards, the exact number of PIWIL2 transcript and miR-146a-3p copies per cell was calculated by comparison of the Ct value to the standard curve.

### Western blotting

Firstly, we extracted protein from cultured cells or samples using RIPA buffer (Sigma, USA). The protein was then separated using SDS-PAGE and transferred onto PVDF membranes (GE, USA). Specific primary antibodies were incubated with the membranes overnight at 4 °C. Subsequently, the membranes were washed thrice and then incubated with secondary antibodies at room temperature for 2 h. Chemiluminescence reagents (Absin, China) were used to visualize the protein bands, which were quantified using Image-Pro Plus 6.0 software (Media Cybernetics, USA) with normalization to GAPDH. The Supplementary Table S3 lists the antibodies used in our research.

### Xenograft tumor models

Balb/c nude mice (18–20 g, 4-week-old males) (n = 75) were obtained from Shanghai Slac Laboratory Animal Co. Ltd. (Shanghai, China) and utilized for the in vivo tumor growth analysis of TPC-1 cells. All mice were housed in a specific pathogen-free conditioned animal care facility with controlled room temperature (22 °C) and normal photoperiods (12 h light/12 h dark). Mice were injected with ketamine (100 mg/kg, i.p.)/acepromazine (5.0 mg/kg, i.p.) for anesthesia. One million TPC-1 cells were subcutaneously injected into the left dorsal flank of each mouse. Tumor growth was measured every 4 days, starting from the fifth day of injection. On the 25th day, an overdose of pentobarbital sodium was used to sacrifice the mice. The tumors were collected and their volume was calculated using the formula (length x width2)/2. The tumor weight was also recorded. All animal experiments were approved by the Ethics Committee of Punan Hospital and were conducted following the National Research Council’s Guide for the Care and Use of Laboratory Animals. The study is reported in compliance with ARRIVE guidelines.

The article "PIWIL2 restrains the progression of thyroid cancer via interaction with miR-146a-3p" was retracted in 2025. Reason: lack of ethics approval or compliance.

### Statistical analysis

The data were processed using statistical software SPSS17.0 (SPSS, Inc., Chicago, IL, USA) and presented as the mean ± S.D. of results obtained from at least three independent experiments. When applicable, a Student t-test was utilized for statistical comparison of continuous data. Pearson’s correlation coefficient was utilized to assess the correlation between the expression of PIWIL2 and miR-146a-3p in TC tissues. Differences between multiple groups were estimated utilizing one-way ANOVA.

## Results

### Negative correlation between the expression of PIWIL2 and miR-146a-3p in TC tissues

Firstly, we collected 20 TC tissue samples and their adjacent tissues to assess the expression levels of PIWIL2 and miR-146a-3p in TC patients. Comparing the adjacent tissues, we found that the mRNA level of PIWIL2 was significantly decreased in TC tissues (P < 0.05), while the level of miR-146a-3p was significantly up-regulated in TC tissues (P < 0.05) (Fig. 1A, B). Linear regression and correlation analyses revealed a negative correlation between the mRNA levels of PIWIL2 and the levels of miR-146a-3p in TC tissues (r2 = 0.6621, P < 0.01) (Fig. 1C). Therefore, when the expression of PIWIL2 decreased, the expression of miR-146a-3p increased. Moreover, we confirmed the down-regulation of PIWIL2 in TC tissues through western blotting (Fig. 1D, E). Our results indicate that PIWIL2 and miR-146a-3p exhibit abnormal expression patterns in TC tissues. The survival times of these 20 patients were monitored and recorded. We classified them into two groups based on their miRNA levels of PIWIL2 and miR-146a-3p, and compared the difference in the survival rates between these two groups. The results are shown in Fig. 1F and G. As depicted in Fig. 1F, the survival rate in the “High PIWIL2” group was significantly different from the “Low PIWIL2” group (P < 0.05). Similarly, the survival rate in the “High miR-146a-3p” group was significantly different from that in the “Low miR-146a-3p” group (P < 0.05) (Fig. 1G).

### PIWIL2 expression was regulated via sponging miR-146a-3p

In light of the negative correlation between miR-146a-3p and PIWIL2 in TC tissues, we conducted further investigations into the association between miR-146a-3p and PIWIL2 in TC cell lines. Firstly, we assessed the expression of miR-146a-3p and PIWIL2 in human normal thyroid follicular epithelial cells (NTHY-ORI 3 − 1) and several TC cell lines. Our findings indicated that the RNA levels of miR-146a-3p and PIWIL2 varied noticeably in TPC-1 or KTC-3 cell lines, particularly TPC-1 cells (Fig. 2A, B).

The article "PIWIL2 restrains the progression of thyroid cancer via interaction with miR-146a-3p" was retracted in 2025. Reason: lack of ethics approval or compliance.

**Fig. 2:** Over-expression of miR-146a-3p down-regulated the expression of PIWIL2 in TC cell lines **(A)** The mRNA level of miR-146a-3p in normal thyroid follicular epithelial cells and various TC cell lines. RNU6B was used for normalization. **(B)** The mRNA level of PIWIL2 in normal thyroid follicular epithelial cells and various TC cell lines. GAPDH was used for normalization. **(C)** The mRNA level of PIWIL2 in TPC-1 cell lines after miR-146a-3p was over-expressed or knocked down. **(D)** The mRNA level of miR-146a-3p in TPC-1 cell lines after miR-146a-3p was over-expressed or knocked down. **E, F.** The protein expression of PIWIL2 in TPC-1 cell lines after miR-146a-3p was over-expressed or knocked down. GAPDH was used for normalization. *: P < 0.05 compared to NTHY-ORI 3 − 1; **: P < 0.01 compared to NTHY-ORI 3 − 1; ^##^: P < 0.01 between groups. N = 6. TC: thyroid cancer

Subsequently, we selected TPC-1 or KTC-3 cell lines for further experiments. In TPC-1 cells, we up-regulated miR-146a-3p expression using a mimic and inhibited gene expression of miR-146a-3p using an inhibitor (Fig. 2D). Our results demonstrated that the expression of PIWIL2 decreased in over-expressed TPC-1 cells of miR-146a-3p and increased after treatment with a miR-146a-3p inhibitor (Fig. 2C, E, F, P < 0.01).

Moreover, we also evaluated the expression of miR-146a-3p in TPC-1 cell lines after over-expression or knocking down of PIWIL2 (Fig. 3A, p < 0.01). Results showed that miR-146a-3p expression decreased in PIWIL2 over-expressed cells and increased in PIWIL2 knocked-down cells (Fig. 3B, P < 0.01).To investigate the underlying mechanism of PIWIL2 and miR-146a-3p in TC, we used absolute quantification to measure the copy number of PIWIL2 and miR-146a in TPC-1 and KTC-3 cell lines. Results are displayed in Fig. 3C. Additionally, we analyzed the pairing relationship between PIWIL2 and miR-146a-3p RNA sequence. Our findings revealed that miR-146a-3p may function as a sponging target of PIWIL2 (Fig. 3D).

**Fig. 3:** The interaction between PIWIL2 and miR-146a-3p in TC cell lines **(A)** The mRNA level of PIWIL2 in TPC-1 cell lines after PIWIL2 was over-expressed or knocked down. **(B)** The mRNA level of miR-146a-3p in TPC-1 cell lines after PIWIL2 was over-expressed or knocked down. **(C)** The copy number of PIWIL2 and miR-146a in TPC-1 and KTC-3 cell lines with absolute quantification. **(D)** The pairing relationship between PIWIL2 and miR-146a-3p RNA sequence. **E, F.** The luciferase activity was tested in 293T cells co-transfected with PIWIL2 WT or PIWIL2 Mut and miR-146a-3p mimic or mimic NC. **G.** The RIP results. ^##^: P < 0.01 between groups. N = 6. TC: thyroid cancer

To validate this hypothesis, we conducted a dual-luciferase reporter assay using a PIWIL2 wild-type reporter construct (PIWIL2-WT) and a mutant PIWIL2-binding site (PIWIL2-Mut). Results showed that miR-146a-3p down-regulated the expression of PIWIL2 in TC cell lines (Fig. 3E, F, P < 0.01). We performed RIP to confirm whether PIWIL2 interacts with miR-146a-3p. Compared to the control group, we found that miR-146a-3p was mostly enriched in the PIWIL2 co-precipitation group (Fig. 3G, P < 0.01).

The article "PIWIL2 restrains the progression of thyroid cancer via interaction with miR-146a-3p" was retracted in 2025. Reason: lack of ethics approval or compliance.

### PIWIL2 and miR-146a-3p modulated cell proliferation, cell cycle progression, and cell apoptosis

The impact of PIWIL2 and miR-146a-3p on cell proliferation was initially examined. The cell proliferation was quantified after over-expressing or knocking down PIWIL2 in TPC-1 and KTC-3 cells with siRNA. Compared to the control group, over-expression of PIWIL2 significantly reduced cell proliferation, but the proliferation was increased after PIWIL2 knockdown (Fig. 4A, B, P < 0.01). The cell proliferation was remarkably increased by up-regulating miR-146a-3p (Fig. 4C, D, P < 0.01). Conversely, inhibiting miR-146a-3p led to a significant inhibition in cell proliferation, (P < 0.01).

**Fig. 4:** Over-expression of miR-146a-3p promoted the proliferation of TC cell lines by down-regulating PIWIL2. **(A)** The cell viability of TPC-1 cells after miR-146a-3p was over-expressed or knocked down. **(B)** The cell viability of TPC-1 cells after PIWIL2 was over-expressed or knocked down. **(C)** The cell viability of KTC-3 cells after miR-146a-3p was over-expressed or knocked down. **(D)** The cell viability of KTC-3 cells after PIWIL2 was over-expressed or knocked down. (**E, F**) The mRNA level of p53 and c-Myc in TPC-1 and KTC-3 cells. (**G**) The protein levels of P21, CyclinD1, PD-1 and CyclinE was measured by Western blot. ^##^: P < 0.01 between groups. N = 6. TC: thyroid cancer

Next, we examined the mRNA levels of cancer-related genes p53 and c-Myc after over-expressing or knocking down PIWIL2 in TPC-1 and KTC-3 cells with siRNA. The results are shown in Fig. 4E and F. PIWIL2 overexpression significantly increased the mRNA levels of anti-cancer gene p53, and PIWIL2 knockdown significantly decreased the mRNA levels of p53 (p < 0.01). In contrast, PIWIL2 overexpression significantly decreased the mRNA levels of pro-cancer gene c-Myc, and PIWIL2 knockdown significantly decreased the mRNA levels of c-Myc (p < 0.01).

We then examined the impact of PIWIL2 and miR-146a-3p on cell cycle progression. Firstly, the expression of CyclinD1, P21, CyclinE, and PD-1 was measured after over-expressing PIWIL2 in TPC-1 and KTC-3 cells (Fig. 4G). PIWIL2 overexpression significantly decreased the expression of CyclinD1, CyclinE, and PD-1, but increased the expression of P21. Over-expressing PIWIL2 led to an increase in the percentage of cells in G0/G1 phase, and a decrease in the percentage of cells in S phase and G2/M phase (Fig. 5A, B, E, P < 0.05). However, miR-146a-3p showed an opposite effect on cell cycle progression. Over-expressing miR-146a-3p decreased the percentage of cells arrested at the G0/G1 phase. Correspondingly, cell numbers in the S phase and G2/M phase significantly increased with miR-146a-3p mimic treatment (Fig. 5C, D, E, P < 0.05). The inhibitor of miR-146a-3p increased the percentage of cells arrested at the G0/G1 phase, but decreased cell numbers in the S phase and G2/M phase (Fig. 5C, D, E, P < 0.05).

The article "PIWIL2 restrains the progression of thyroid cancer via interaction with miR-146a-3p" was retracted in 2025. Reason: lack of ethics approval or compliance.

**Fig. 5:** Over-expression of miR-146a-3p changed the cell cycle of TC cell lines by down-regulating PIWIL2. **(A)** The cell cycle of TPC-1 cells after miR-146a-3p was over-expressed or knocked down. **(B)** The cell cycle of TPC-1 cells after PIWIL2 was over-expressed or knocked down. **(C)** The cell cycle of KTC-3 cells after miR-146a-3p was over-expressed or knocked down. **(D)** The cell cycle of KTC-3 cells after PIWIL2 was over-expressed or knocked down. **(E)** The flow cytometry analysis of cell cycle of TPC-1 cells. ^#^: P < 0.05 between groups. N = 6. TC: thyroid cancer

Finally, we evaluated the impact of PIWIL2 and miR-146a-3p on the apoptosis of TC cells. PIWIL2 overexpression dramatically promoted cell apoptosis (Fig. 6A, B, E, P < 0.01). After treatment with miR-146a-3p mimic, apoptosis in TPC-1 and KTC-3 cells was inhibited, but the apoptosis was reversed by miR-146a-3p inhibitor treatment (Fig. 6C, D, E, P < 0.01).

**Fig. 6:** PIWIL2 and miR-146a-3p regulated the apoptosis of TC cell lines **(A)** The apoptosis of TPC-1 cells after over-expressed miR-146a-3p or knockdown miR-146a-3p. **(B)** The apoptosis of TPC-1 cells after over-expressed PIWIL2 or knockdown PIWIL2. **(C)** The apoptosis of KTC-3 cells after over-expressed miR-146a-3p or knockdown miR-146a-3p. **(D)** The apoptosis of KTC-3 cells after over-expressed PIWIL2 or knockdown PIWIL2. **(E)** The flow cytometry analysis of apoptosis of TPC-1 cells after over-expressed miR-146a-3p, knockdown miR-146a-3p, over-expressed PIWIL2 or knockdown PIWIL2. ^##^: P < 0.01 between groups. N = 6. TC: thyroid cancer

### miR-146a-3p and PIWIL2 affected the migration and invasion of TC cells

The wound healing assay demonstrated that miR-146a-3p significantly increased TPC-1 cell invasion when compared to the Control group (Fig. 7A, P < 0.01). Similarly, the transwell assay suggested that miR-146a-3p significantly upregulated the cell invasion in TPC-1 cells (Fig. 7B, P < 0.01). Conversely, the overexpression of PIWIL2 significantly inhibited the invasion of TPC-1 cells when compared to the siRNA and Control groups (Fig. 7C, P < 0.01). Moreover, the upregulation of PIWIL2 reduced TPC-1 cell invasion (Fig. 7D, P < 0.01). These experiments confirmed that miR-146a-3p increased the migration and invasion abilities of TPC-1 cells, while PIWIL2 inhibited them.

The article "PIWIL2 restrains the progression of thyroid cancer via interaction with miR-146a-3p" was retracted in 2025. Reason: lack of ethics approval or compliance.

**Fig. 7:** miR-146a-3p and PIWIL2 regulated the migration and invasion of TC cell lines **(A)** The migration of TPC-1 cells after miR-146a-3p was overexpressed or knocked down. **(B)** The invasion of TPC-1 cells after miR-146a-3p was overexpressed or knocked down. **(C)** The migration of TPC-1 cells after PIWIL2 was overexpressed or knocked down. **(D)** The invasion of TPC-1 cells after PIWIL2 was overexpressed or knocked down.   ^#^: P<0.05 between groups;  ^##^: P < 0.01 between groups. N = 6. TC: thyroid cancer

### PIWIL2 and miR-146a-3p affected the progression of TC in nude mice

The role of miR-146a-3p and PIWIL2 in thyroid cancer (TC) was further validated through the use of a xenograft tumor model. In comparison to the Control group, xenograft tumor mice injected with over-expressed PIWIL2 cells showed a lightened body weight, lower percent survival, smaller tumor size, and reduced tumor weight (Fig. 8A-E, P < 0.01). Conversely, inhibiting PIWIL2 increased the percent survival and decreased the body weight, tumor size, and weight of the xenograft animal model. The pathological effects of miR-146a-3p were opposite, where xenograft tumor mice treated with miR-146a-3p mimic showed an increased body weight, a higher percent survival, larger tumor size, and weight (Fig. 9A-D, P < 0.01). On the other hand, miR-146a-3p inhibitor decreased percent survival and increased the body weight, tumor size, and weight of xenograft animal models.

**Fig. 8:** PIWIL2 regulated the progression of TC animal models **(A)** The body weight of mice after mice were injected with TC cells with over-expressed PIWIL2 or knockdown PIWIL2. **(B)** The survival percent of mice after mice were injected with TC cells with over-expressed PIWIL2 or knockdown PIWIL2. **(C)** The tumor size of xenograft tumor after mice were injected with TC cells with over-expressed PIWIL2 or knockdown PIWIL2. **(D)** The tumor weight of xenograft tumor after mice were injected with TC cells with over-expressed PIWIL2 or knockdown PIWIL2. **(E)** The image of xenograft tumor after mice were injected with TC cells with over-expressed PIWIL2 or knockdown PIWIL2. ^##^: P < 0.01 between groups. N = 6. TC: thyroid cancer

**Fig. 9:** miR-146a-3p regulated the progression of TC animal models **(A)** The body weight of mice after mice were injected with TC cells with over-expressed miR-146a-3p or knockdown miR-146a-3p. **(B)** The survival percent of mice after mice were injected with TC cells with over-expressed miR-146a-3p or knockdown miR-146a-3p. **(C)** The tumor size of xenograft tumor after mice were injected with TC cells with over-expressed miR-146a-3p or knockdown miR-146a-3p. **(D)** The tumor weight of xenograft tumor after mice were injected with TC cells with over-expressed miR-146a-3p or knockdown miR-146a-3p. ^##^: P < 0.01 between groups. N = 6. TC: thyroid cancer

To confirm the effects of miR-146a-3p-modulated PIWIL2 on thyroid tumorigenesis in vivo, rescue tests were executed using a xenograft tumor mice model. Results showed that down-regulation of miR-146a-3p triggered a distinct suppression on TC progression, which could be recovered by PIWIL2 siRNA injection (Fig. 10A-D, P < 0.01). As expected, over-expressed PIWIL2 injection reversed the effects of miR-146a-3p over-expression on amplifying tumor size and weight of xenograft tumors (P < 0.01). Collectively, it supports that both PIWIL2 and miR-146a-3p are involved in the progression of TC in vivo.

The article "PIWIL2 restrains the progression of thyroid cancer via interaction with miR-146a-3p" was retracted in 2025. Reason: lack of ethics approval or compliance.

**Fig. 10:** PIWIL2 regulated the progression of TC animal models via miR-146a-3p **(A)** The body weight of mice after injected over-expressed PIWIL2 and knockdown miR-146a-3p or knockdown PIWIL2 and over-expressed miR-146a-3p TC cells. **(B)** The survival percent of mice after injected over-expressed PIWIL2 and knockdown miR-146a-3p or knockdown PIWIL2 and over-expressed miR-146a-3p TC cells. **(C)** The tumor size of xenograft tumor after injected over-expressed PIWIL2 and knockdown miR-146a-3p or knockdown PIWIL2 and over-expressed miR-146a-3p TC cells. **(D)** The tumor weight of xenograft tumor after injected over-expressed PIWIL2 and knockdown miR-146a-3p or knockdown PIWIL2 and over-expressed miR-146a-3p TC cells. ^##^: P < 0.01 between groups. N = 6. TC: thyroid cancer

## Discussion

TC is the most common and pervasive endocrine malignancy, particularly in women [10]. From 1990 to 2021, the incidence and mortality rates of TC have been consistently increasing [11]. In developed countries, there are currently up to 586,202 newly diagnosed cases and 43,646 deaths according to the estimates from Global Cancer Statistics in 2020 [15]. Thanks to early detection and optimal treatments, the survival rate of differentiated TCs has significantly improved. Patients with early stage DTCs have a 5-year survival rate approaching 98% and a recurrence rate of less than 5–10% [16, 17]. However, the prognosis for advanced-stage TC cases or those with multiple organ metastasis remains poor, with a 5-year survival rate of only 15.3% [18]. It is therefore essential to further elucidate the pathological mechanisms of TC.

The article "PIWIL2 restrains the progression of thyroid cancer via interaction with miR-146a-3p" was retracted in 2025. Reason: lack of ethics approval or compliance.

In the present study, we found that PIWIL2 and miR-146a-3p exhibited aberrant expression in TC tissues. Compared with para-carcinoma tissues, TC tissues showed low expression of PIWIL2 and high expression of miR-146a-3p. We also uncovered a specific mechanism in which PIWIL2 acts as a sponge for miR-146a-3p, inhibiting the progression of TC in vivo and in vitro. These findings suggest that PIWIL2 and miR-146a-3p could serve as therapeutic or diagnostic targets for TC.

PIWIL2, a piRNA binding protein that is essential for testicular reproductive function, has been found to be involved in human malignancies, such as lung, breast, colon, prostate, and cervix cancers. However, despite conflicting expression alterations found in the GEPIA2 database [19] [20], the role of PIWIL2 in TC has not yet been revealed. In this study, we found that the mRNA and protein levels of PIWIL2 were significantly lower in TC tissues and cell lines compared to the counterparts. This result is consistent with TCGA data, although a previous study reported a significant up-regulation of protein expression levels of PIWIL2 in papillary and micropapillary thyroid cancers, while mRNA expression changes were statistically insignificant [20]. It’s a very complicated thing when it comes to clinical samples. There are many factors affecting clinical samples, for example, unknown coexisting diseases, sudden mental stress, sampling chance, and so on. We proposed that this discrepancy may be due to the distinctive stage, race, sampling chance, and sample size of thyroid cancers.

We also demonstrated that down-regulated PIWIL2 may promote the proliferation and metastasis of TC cells in vitro. We found that PIWIL2 overexpression increased the mRNA levels of anti-cancer gene p53, while PIWIL2 siRNA decreased the mRNA levels of p53. Conversely, PIWIL2 overexpression decreased the mRNA levels of pro-cancer gene c-Myc, while PIWIL2 siRNA decreased the mRNA levels of c-Myc. Moreover, PIWIL2 overexpression decreased the expression of CyclinD1, CyclinE, and PD-1 but increased the expression of P21. In vivo experiments using a xenograft tumor model also showed that PIWIL2 may inhibit the progression of TC. These findings suggest that PIWIL2 plays a significant role in the pathogenesis of TC.

MiR-146a-3p has been reported to be a crucial factor in various types of cancers. For instance, it may regulate the expression of PTTG1, thereby promoting the growth, invasion, metastasis, and migration of bladder cancer [21]. In prostate cancer, miRNA-146a-3p targeting APIP regulates cell growth and migration via the ERK1/2 pathway and is a promising biomarker [22]. However, its exact role in TC is largely unknown. Our study aims to identify the detailed role of miR-146a-3p in TC. Our findings reveal that miR-146a-3p is up-regulated in TC tissues and is responsible for promoting the proliferation, invasion, and migration of TC cells, while inhibiting their apoptosis. We observed a decrease in PIWIL2 expression in miR-146a-3p over-expressed TPC-1 cells, which increased after treatment with miR-146a-3p inhibitor. Conversely, the expression of miR-146a-3p decreased in PIWIL2 over-expressed cells and increased in PIWIL2 knocked-down cells. Our RNA sequence analysis suggests that miR-146a-3p may be a sponging target of PIWIL2. Dual-luciferase reporter assay confirmed that miR-146a-3p down-regulates the expression of PIWIL2 in TC cell lines. Furthermore, RIP results showed that miR-146a-3p was mainly enriched in the PIWIL2 co-precipitation group, indicating that PIWIL2 directly interacts with miR-146a-3p. The xenograft tumor model confirmed the role of miR-146a-3p in the progression of TC, suggesting that it may promote the advancement of TC.

The article "PIWIL2 restrains the progression of thyroid cancer via interaction with miR-146a-3p" was retracted in 2025. Reason: lack of ethics approval or compliance.

Our study suggests that PIWIL2 may sponge miR-146a-3p to modulate the proliferation, invasion, migration, and apoptosis of TC cells. As PIWIL2 and miR-146a-3p are crucial factors in the development of TC, they may be potential therapeutic targets for TC treatment in the early stages, recrudescence treatment, and metastasis treatment. Additionally, miR-146a-3p may serve as a new biomarker of TC, as it can be detected in different body fluids. However, the detailed molecular mechanism underlying the role of miR-146a-3p in TC remains to be elucidated.

## Conclusion

Despite the classical role of PIWIL2 in mediating reproduction by binding to piRNA, we have uncovered its role in the development of TC. We identified opposite expression alterations of PIWIL2 and miR-146a-3p in TC tissues and determined that PIWIL2 may act as a ‘sponge’ by adsorbing miR-146a-3p, which leads to inhibition of proliferation, metastasis, and cell cycle progression, while decelerating apoptosis of TC cells. In short, PIWIL2 serving as a sponge for miR-146a-3p, illuminating a new role of PIWIL2 distinguished from its classical role by binding to piRNA.

## Electronic supplementary material

Below is the link to the electronic supplementary material.

Supplementary Material 1

Supplementary Material 2

Supplementary Material 3

Supplementary Material 4

Supplementary Material 5

Supplementary Material 6

Supplementary Material 7

The article "PIWIL2 restrains the progression of thyroid cancer via interaction with miR-146a-3p" was retracted in 2025. Reason: lack of ethics approval or compliance.

## Data Availability

The datasets used and/or analyzed for this study are available from the corresponding author upon reasonable request.
